The article "Munro Pressure Ulcer Risk Assessment Scale in Adult Patients Undergoing General Anesthesia in the Operating Room" was published in 2022. Journal: J Healthc Eng.

# Munro Pressure Ulcer Risk Assessment Scale in Adult Patients Undergoing General Anesthesia in the Operating Room

**DOI:** 10.1155/2022/4157803

**Published:** 2022-03-21

**Authors:** Lumin Lei, Ti Zhou, Xinlin Xu, Lihong Wang

**Affiliations:** ^1^Department of Anesthesiology, The Fourth Medical Center of PLA Central Hospital, Beijing 100048, China; ^2^Operating Room, People's Hospital of Hengshui City, Hebei Province, Hengshui 053000, China

## Abstract

Pressure ulcers are a common complication of immobility and frequently occur in surgical patients. The occurrence of pressure ulcers is affected by many factors, such as operation time and position, anesthesia method, and postoperative nursing. The aim of this study was to investigate the Munro Pressure Ulcer Risk Assessment Scale's value in predicting acute pressure ulcers in general anesthesia patients. This case-control study included patients who underwent more than 2 hours of general anesthesia in our hospital from January 2018 to December 2020. The case group comprised 42 patients who had pressure sores in surgical compression sites within 3 days after surgery. The control group consisted of 84 patients without acute pressure sores after surgery. Baseline patient data were compared between the two groups, and a logistic multivariate model was used to analyze potential risk factors for acute pressure ulcers. The Munro Pressure Ulcer Risk Assessment Scale scores and Braden scale scores were compared between the two groups during and after surgery. A receiver operating characteristic curve was used to evaluate the clinical value of the two scales (administered at the two time points) in predicting the occurrence of acute pressure ulcers after surgery. The operation and anesthesia times of patients in the case group were longer than those in the control group (*P* < 0.05). The proportion of comatose patients and patients with diabetes were significantly higher in the case group. While the case group had higher Munro scores during and after surgery compared to the control group (*P* < 0.05), Braden scores at the corresponding time points were lower (*P* < 0.05). The following variables were identified as independent risk factors of acute pressure ulcers: prolonged operation time and anesthesia time, increase in Munro scores during and after operation, decrease in Braden scores during and after operation, and comatose status (*P* < 0.05). The area under the receiver operating characteristic curve (AUC) of the postoperative Munro score for predicting postoperative pressure ulcer risk was 0.774; the sensitivity and specificity were 67.73% and 80.58%, respectively. The AUC of the intraoperative Braden score for predicting postoperative pressure ulcer risk was 0.836, with a sensitivity of 78.95% and specificity of 78.00%. The AUC of the postoperative Braden score for predicting postoperative pressure ulcer risk was 0.809, with a sensitivity of 73.58% and specificity of 64.26% (*P* < 0.05). Our results indicate that the intraoperative Munro Pressure Ulcer Risk Assessment Scale is highly effective for predicting the risk of postoperative pressure ulcers in surgical patients who require general anesthesia.

The article "Munro Pressure Ulcer Risk Assessment Scale in Adult Patients Undergoing General Anesthesia in the Operating Room" was published in 2022. Journal: J Healthc Eng.

## 1. Introduction

Pressure ulcers are localized areas of skin damage that may also involve the subcutaneous soft tissues. They generally occur over bony prominences and in areas where there is contact between the skin and medical equipment. Recent studies have reported a high incidence of pressure ulcers in surgical patients. There are a wide range of risk factors for surgical pressure ulcers, including patient physiological and pathological factors, operative factors, anesthesia-related complications, and the use of various instruments. The clinical prevention of pressure ulcers is based on the professional and standardized assessment of patients and the provision of adequate protection [1].

While there is currently a wide range of risk assessment scales for pressure ulcers, the Braden scale is the most used measure in China and abroad. However, some studies have indicated that this scale has a limited ability to predict ulcer risk in different populations and clinical environments. The Munro Pressure Ulcer Risk Assessment Scale is the first pressure ulcer scale to be specifically developed for surgical patients. However, its use is relatively cumbersome due to the large number of assessment items and the need for some items to be evaluated with the assistance of anesthesiologists. As a result, the Munro Pressure Ulcer Risk Assessment Scale is not widely used in the clinic [2]. In order to investigate the clinical value of the adult version of this scale, we compared its scores with those of the Braden scale during and after surgeries in patients requiring general anesthesia. We also compared the ability of these two scales to predict postoperative pressure ulcer risk.

## 2. Materials and Methods

### 2.1. General Information

This case-control study included patients who underwent more than 2 h of general anesthesia in our hospital from January 2018 to December 2020. The case group comprised 42 patients who developed pressure sores at a compression site within 3 days after surgery. The control group included 84 patients without acute pressure sores after surgery.

Inclusion criteria were as follows: operations with a duration of ≥2 h that were performed under general anesthesia; evaluation with both the Munro Pressure Ulcer Risk Assessment Scale and Braden scale at the end of surgery and after patient departure from the anesthesia observation room, patient age ranging from 19 to 75 years, pressure sores appearing at a compression site within 72 h after the operation and diagnosed according to the criteria of the Prevention and Treatment Guidelines for Pressure Sores (2014 edition), and provision of written informed consent. The study protocol was approved by the Medical Ethics Committee of our institution. The exclusion criteria consisted of the following: presence of preoperative pressure ulcers and skin ulcers, posture changes during the operation, posture duration of <2 h, patients under local anesthesia, and other relevant factors affecting this study.

The article "Munro Pressure Ulcer Risk Assessment Scale in Adult Patients Undergoing General Anesthesia in the Operating Room" was published in 2022. Journal: J Healthc Eng.

### 2.2. Pressure Ulcer Assessment Scales

The intraoperative Munro Pressure Ulcer Risk Assessment Scale [3] includes the following components: anesthesia classification, anesthesia method, intraoperative body temperature, hypotension, skin humidity, posture change during surgery, and surgical posture. A total score of ≤13 indicates a low risk for pressure ulcers. The postoperative Munro Pressure Ulcer Risk Assessment Scale mainly evaluates operation time and blood loss. A total score of ≤15 indicates a low risk for pressure ulcers.

The Braden scale [4] includes six assessment categories. These include the patients' sensory perceptions, degree of mobility, nutrition status, activity level, exposure to moisture, and degree of friction and shear force upon movement. The maximum score is 23, with lower scores indicating a higher risk of postoperative acute pressure ulcers. A score of ≤14 reflects a medium to high risk for pressure ulcers.

The investigators in this study were nurses at our hospital. All investigators had at least 3 years of clinical work experience and had undergone a 2-week online training program. The training content included the definition and staging criteria for pressure ulcers, pressure ulcer pathophysiology and risk factors, instructions on how to use the pressure ulcer assessment scales, precautions, and preventive measures for pressure ulcers. The two pressure ulcer scale assessments were conducted by two evaluators at different times. Simultaneously, the evaluators maintained double blindness to avoid deviation. The skin condition of the patients was carefully examined before and after the operation. The characteristics of the pressure ulcers were recorded in detail upon detection. The following patient data were extracted from our hospital's computer system: age, sex, body mass index, smoking and drinking status, and combined with chronic diseases and surgical conditions.

The article "Munro Pressure Ulcer Risk Assessment Scale in Adult Patients Undergoing General Anesthesia in the Operating Room" was published in 2022. Journal: J Healthc Eng.

### 2.3. Statistical Analysis

The distribution of the Munro Pressure Ulcer Risk Assessment Scale and Braden scale scores were tested for normality (expressed as $\bar{X}\pm s$). The *t*-test was used to compare mean scores between the two groups. Enumeration data are presented as counts and percentages (*n* (%)). Comparisons of categorical variables (e.g., complication rate, sex, and comorbidities between groups were performed with the *χ*^2^ test. A multivariate analysis was conducted using a conditional logistic regression model, and the predictive model was evaluated using receiver operating characteristic (ROC) curve analysis. All statistical analyses were performed with the SPSS 21.0 software program. The level of statistical significance was set at *α* = 0.05.

## 3. Results

### 3.1. Results of Single Factor Analysis

First, the *t*-test and *χ*2 test were used to analyze the factors of postoperative acute pressure ulcer in the case group and the control group. The results showed age, BMI, gender, smoking, drinking, hypertension, hyperlipidemia, and surgical type were compared between the case group and the control group, and the difference was not statistically significant (*P* > 0.05). The operation time and anesthesia time in the case group were longer than those in the control group (*P* < 0.05). The Munro scores during and after operation, the proportion of coma patients, and the proportion of patients with diabetes in the case group were higher than those in the control group (*P* < 0.05). The Braden scores during and after operation in the case group were lower than those in the control group (*P* < 0.05).  Table 1 provides the results of single factor analysis.

### 3.2. Multivariate Analysis Results of Acute Pressure Ulcers after Surgery

The occurrence of acute pressure ulcer within 3 days after operation was taken as the dependent variable, and the operation time, anesthesia time, intraoperative and postoperative Munro scores, the proportion of coma patients, the prevalence rate of diabetes, and intraoperative and postoperative Braden scores were taken as independent variables by univariate analysis. The results showed that prolonged operation and anesthesia time, the increase of intraoperative and postoperative Munro scores, decreased intraoperative and postoperative Braden scores, and coma in patients after general anesthesia were independent risk factors for the occurrence of acute pressure ulcer after general anesthesia (*P* < 0.05).  Table 2 provides multivariate analysis results of acute pressure ulcers after surgery.

### 3.3. Intraoperative and Postoperative Munro Score and Braden Score Predict ROC Curve Analysis Results of Pressure Ulcers in Patients Undergoing General Anesthesia

ROC curves were drawn for intraoperative and postoperative Munro score and intraoperative and postoperative Braden score. The results showed that the area under the ROC curve (AUC) value of intraoperative Munro score in predicting the risk of postoperative pressure ulcer in patients undergoing general anesthesia was 0.874, the sensitivity was 85.92%, and the specificity was 78.41%. The AUC value of postoperative Munro score in predicting the risk of postoperative pressure ulcer in patients undergoing general anesthesia was 0.774, the sensitivity was 67.73%, and the specificity was 80.58%. The AUC value of intraoperative Braden score in predicting the risk of postoperative pressure ulcer in patients undergoing general anesthesia was 0.836, the sensitivity was 78.95%, and the specificity was 78.00%. The AUC value of postoperative Braden score in predicting the risk of postoperative pressure ulcer in patients undergoing general anesthesia was 0.809, the sensitivity was 73.58%, and the specificity was 64.26% (*P* < 0.05).  Table 3 provides ROC curve analysis results of Munro scores and Braden scores predicting pressure ulcers in patients undergoing general anesthesia during and after surgery.  Figure 1 shows the ROC curve of Munro score and Braden score predicting the occurrence of pressure ulcers in patients during operation.  Figure 2 shows the ROC curve of Munro score and Braden score predicting the occurrence of pressure ulcers in patients after surgery.

The article "Munro Pressure Ulcer Risk Assessment Scale in Adult Patients Undergoing General Anesthesia in the Operating Room" was published in 2022. Journal: J Healthc Eng.

## 4. Results Analysis

Pressure ulcers frequently occur perioperatively and have a serious impact on postoperative care and patient recovery. At present, the structured assessment of pressure ulcer risk remains the primary method for facilitating the formulation of preventive measures. Therefore, it is pertinent that the tools selected for pressure ulcer risk assessment are accurate and reliable [5]. Some studies have reported that the occurrence of pressure ulcers in the perioperative period is related to patient, surgical, and anesthesia factors, which are associated with the entirety of the patient. The assessment of preoperative risk factors for pressure ulcers does not account for risk factors that become evident during the surgical procedure. Likewise, the restriction of pressure ulcer risk assessment to intraoperative factors does not account for postoperative risk factors. Therefore, it is recommended that risk factors for pressure ulcers be continually evaluated over the entire hospitalization and recovery period [6].

In the present study, we found that both the operation and anesthesia time were longer in patients with pressure ulcers compared to those in the control group. While patients with pressure ulcers had higher Munro Pressure Ulcer Risk Assessment Scale scores during and after surgery compared to the control group, Braden scores at the corresponding time points were lower. These results indicate that pressure ulcer occurrence was related to the operation time and anesthesia time. At the same time, patients with diabetes were more prone to pressure ulcers, and Munro scores during and after surgery were relatively high. Longer operation and anesthesia times result in prolonged skin tissue compression and ischemia-hypoxia time during the perioperative period. Indeed, it has been previously reported that the incidence of tooth trauma in patients with operation times exceeding 4 h increases by 33% every 30 min [7–9]. Some investigators have suggested that operation time is proportional to the risk of pressure ulcers, which also indicates an increase in the risk of operation. Therefore, the risk of pressure ulcers may be reduced by ensuring sufficient preoperative planning; this would in turn facilitate a smooth surgical workflow and shorten the operation time as much as possible [10–12].

The article "Munro Pressure Ulcer Risk Assessment Scale in Adult Patients Undergoing General Anesthesia in the Operating Room" was published in 2022. Journal: J Healthc Eng.

Diabetes was more prevalent among patients with pressure ulcers. This result is supported by a prior study that reported that pressure ulcer risk was three times higher in diabetic patients compared to nondiabetic patients [13–15]. A continuous increase in blood glucose reduces oxygen supply in human tissues. This delays reactive hyperemia during the operation and accelerates vascular occlusion.

This study compared the use of the Braden scale and Munro Pressure Ulcer Risk Assessment Scale in perioperative patients. While the Braden scale is the most commonly used tool for evaluating pressure ulcers in clinical practice, some studies have reported that it is only suitable for hospitalized bedridden patients and the elderly. The universal assessment scale lacks items that pertain to specific risk factors; it therefore has a low predictive value for pressure ulcers and is unable to provide a comprehensive evaluation of pressure ulcer risk [16]. Some studies have shown that patients cannot be evaluated for the pressure ulcer risk factors in the process of operation after surgery, but only take the surgical patients as ordinary inpatients for pressure ulcer risk assessment [17]. The Munro Pressure Ulcer Risk Assessment Scale (adult version) is used to assess the risk of pressure ulcers during the perioperative period, which can be divided into preoperative, intraoperative, and postoperative periods to facilitate patient evaluation. The advantages of this scale are that it can provide an initial evaluation of pressure ulcer risk before surgery, and it can also be continuously used in follow-up assessments during the postoperative period, until hospital discharge [18].

The article "Munro Pressure Ulcer Risk Assessment Scale in Adult Patients Undergoing General Anesthesia in the Operating Room" was published in 2022. Journal: J Healthc Eng.

ROC curve analysis in the present study indicated that the AUC of the intraoperative Munro Pressure Ulcer Risk Assessment Scale score for predicting the risk of postoperative pressure ulcers was 0.874, with a sensitivity and specificity of 85.92% and 78.41%, respectively. The AUC of the postoperative Munro Pressure Ulcer Risk Assessment Scale score was lower than that for the Braden scale. The AUC is one of the most comprehensive indicators of prediction accuracy. The high validity and accuracy of the Munro Pressure Ulcer Risk Assessment Scale may be attributed to its incorporation of both intraoperative and postoperative items that are completed by operating room nurses and anesthesiologists. Braden scale items reflect the mechanism of stress injury and do not account for the unique risk factors inherent to surgical patients [19].

Sensitivity and specificity were also assessed in the present study. Sensitivity, also referred to as the true positive rate, is the ability of a test to correctly identify patients with a disease. Thus, it can be used to indicate the ability of a scale to predict surgically acquired stress injuries. Specificity, also referred to as the true negative rate, is the ability of a test to correctly identify patients without a disease. It can therefore be used to predict which cases will be unaffected by surgically acquired stress injuries. High sensitivity and specificity are considered to be the most important attributes of an evaluation scale. The high sensitivity of the Munro Pressure Ulcer Risk Assessment Scale makes it particularly effective as a screening test for identifying patients at risk of surgically acquired stress injuries, as well as a guide for the implementation of preventive measures by nurses.

## 5. Conclusion

In the present study, we assessed the ability of the Munro Pressure Ulcer Risk Assessment Scale to rapidly and accurately predict the risk of pressure ulcers in patients under general anesthesia. This scale is the only assessment tool for pressure ulcers that can be used continuously throughout the entirety of the perioperative period. By comparing its reliability, validity, advantages, disadvantages, and predictive ability with that of the more commonly used Braden scale, we have demonstrated that the Munro Pressure Ulcer Risk Assessment Scale warrants consideration for widespread use in operating rooms in China. However, some limitations are acknowledged in the present study. First, this study did not refine the types of surgery, which may lead to limitations in data collection. Second, some patients may have used other preventive measures for pressure ulcers; this may have resulted in a low incidence of pressure ulcers, thus affecting the accuracy of the research results. Therefore, additional studies with larger sample sizes are warranted to confirm the reliability, validity, practicability, and effectiveness of the Munro Pressure Ulcer Risk Assessment Scale.

The article "Munro Pressure Ulcer Risk Assessment Scale in Adult Patients Undergoing General Anesthesia in the Operating Room" was published in 2022. Journal: J Healthc Eng.

In summary, the Munro Pressure Ulcer Risk Assessment Scale was used to evaluate the risk of pressure ulcers in general anesthesia patients during and after surgery. The results indicated that the intraoperative Munro Pressure Ulcer Risk Assessment Scale score is highly effective for predicting the risk of postoperative pressure ulcers in this patient group [20, 21].

## Figures and Tables

**Figure 1:** The ROC curve of Munro score and Braden score predicting the occurrence of pressure ulcers in patients during operation.

**Figure 2:** The ROC curve of Munro score and Braden score predicting the occurrence of pressure ulcers in patients after surgery.

**Table 1:** Results of single factor analysis.

Factor	Case group (*n* = 42)	Control group (*n* = 84)	*t*/*χ*^2^	*P*
Age (year)	50.9 ± 8.1	49.5 ± 7.8	0.938	0.350
BMI (kg/m^2^)	24.8 ± 2.2	24.2 ± 2.0	1.535	0.127
Operation time (min)	159.2 ± 18.7	152.0 ± 15.5	2.291	0.024
Anesthesia time (min)	177.2 ± 19.4	166.8 ± 18.5	2.927	0.004
Intraoperative Munro score (points)	18.49 ± 3.11	14.37 ± 3.04	7.117	0.000
Postoperative Munro score (points)	16.28 ± 3.30	13.82 ± 2.95	4.240	0.000
Intraoperative Braden score (points)	10.14 ± 2.50	14.32 ± 2.87	−8.034	0.000
Postoperative Braden score (points)	11.04 ± 2.67	14.54 ± 2.72	−6.850	0.000
Gender (%)			1.029	0.301
Male	26 (61.9)	44 (52.38)		
Female	16 (38.1)	40 (47.62)		
Smoking (%)			1.289	0.256
Yes	14 (33.33)	20 (23.81)		
No	28 (66.67)	64 (76.19)		
Drinking (%)			0.197	0.657
Yes	11 (26.19)	19 (22.62)		
No	31 (73.81)	65 (77.38)		
Hypertension (%)			0.871	0.377
Yes	22 (52.38)	37 (44.05)		
No	20 (47.62)	47 (55.95)		
Diabetes (%)			6.074	0.011
Yes	11 (26.19)	8 (9.52)		
No	31 (73.81)	76 (90.48)		
Hyperlipidemia (%)			0.969	0.325
Yes	14 (33.33)	21 (25)		
No	28 (66.67)	63 (75)		
Type of surgery (%)			2.705	0.608
Orthopedics	8 (19.05)	14 (16.67)		
General surgery	4 (9.52)	15 (17.86)		
Cardiothoracic surgery	11 (26.19)	24 (28.57)		
Neurosurgery	15 (35.71)	21 (25)		
Others	4 (9.52)	10 (11.9)		
Coma (%)			6.074	0.011
Yes	11 (26.19)	8 (9.52)		
No	31 (73.81)	76 (90.48)		

**Table 2:** Multivariate analysis results of acute pressure ulcers after surgery.

Factor	*β*	SE	Wald's	*P*	OR	95% CI	
Intraoperative Munro score (points)	0.718	0.271	7.020	0.001	2.050	1.205	3.487
Postoperative Munro score (points)	0.664	0.264	6.326	0.005	1.943	1.158	3.259
Intraoperative Braden score (points)	0.593	0.257	5.324	0.032	1.809	1.093	2.994
Postoperative Braden score (points)	0.577	0.265	4.741	0.044	1.781	1.059	2.993
Operation time (min)	0.498	0.227	4.813	0.042	1.645	1.055	2.567
Anesthesia time (min)	0.477	0.231	4.264	0.048	1.611	1.025	2.534
Diabetes	0.617	0.452	1.863	0.227	1.853	0.764	4.495
Coma	0.485	0.221	4.816	0.042	1.624	1.053	2.505
Constant term	1.102	0.595	3.430	0.093	3.010	0.938	9.662

The article "Munro Pressure Ulcer Risk Assessment Scale in Adult Patients Undergoing General Anesthesia in the Operating Room" was published in 2022. Journal: J Healthc Eng.

**Table 3:** ROC curve analysis results of Munro scores and Braden scores predicting pressure ulcers in patients undergoing general anesthesia during and after surgery.

Factor	Cutoff value	Sensitivity (%)	Specificity (%)	Missed diagnosis rate (%)	Misdiagnosis rate (%)	AUC
Intraoperative Munro score (points)	16.20	85.92	78.41	14.08	21.59	0.874
Postoperative Munro score (points)	15.71	67.73	80.58	32.27	19.42	0.774
Intraoperative Braden score (points)	10.28	78.95	78.00	21.05	22.00	0.836
Postoperative Braden score (points)	10.76	73.58	64.26	26.42	35.74	0.809

## Data Availability

The data used to support the findings of this study are available from the corresponding author upon request.
